# Comparative Study on Plant Latex Particles and Latex Coagulation in *Ficus benjamina*, *Campanula glomerata* and Three *Euphorbia* species

**DOI:** 10.1371/journal.pone.0113336

**Published:** 2014-11-19

**Authors:** Georg Bauer, Stanislav N. Gorb, Marie-Christin Klein, Anke Nellesen, Max von Tapavicza, Thomas Speck

**Affiliations:** 1 Plant Biomechanics Group, Botanic Garden, Faculty of Biology, University of Freiburg, Freiburg, Germany; 2 FMF – Freiburg Materials Research Center, University of Freiburg, Freiburg, Germany; 3 Functional Morphology and Biomechanics, Zoological Institute, University of Kiel, Kiel, Germany; 4 Fraunhofer Institute for Environmental, Safety, and Energy Technology UMSICHT, Oberhausen, Germany; Massey University, New Zealand

## Abstract

Among latex-producing plants, mainly the latex of *Hevea brasiliensis* has been studied in detail so far, while comprehensive comparative studies of latex coagulation mechanisms among the more than 20,000 latex-bearing plant species are lacking. In order to give new insights into the potential variety of coagulation mechanisms, the untreated natural latices of five latex-bearing plants from the families Euphorbiaceae, Moraceae and Campanulaceae were visualised using Cryo-SEM and their particle size compared using the laser diffraction method. Additionally, the laticifers of these plants species were examined *in planta* via Cryo-SEM. Similar latex particle sizes and shape were found in *Ficus benjamina* and *Hevea brasiliensis*. Hence, and due to other similarities, we hypothesize comparable, mainly chemical, coagulation mechanisms in these two species, whereas a physical coagulation mechanism is proposed for the latex of *Euphorbia* spp. The latter mechanism is based on the huge amount of densely packed particles that after evaporation of water build a large surface area, which accelerates the coagulation procedure.

## Introduction

Latex, a sticky sap that flows out of some plants upon wounding, can be found in more than 20 000 species from some 40 families [1], [2]. It is stored in laticifers (specialized cells or chains of cells containing latex [3]) and seals wounds as it coagulates when discharged from those. Besides the simple sealing of the wound, latex functions range from a plant defense system to the restoration of the mechanical properties of injured plants [2], [4], [5], [6]. Not only the latices differ interspecifically, e.g. in their colour and chemical composition [5], but also different types of laticifers can be found (Figure 1). Some species like *Hevea brasiliensis* are equipped with articulated laticifers that are composed of chains of cells joined together. Such chains can be unbranched (non-anastomosing) or laterally connected, thus forming a net-like structure (anastomosing). The laticifers of other plants like *Ficus benjamina* consist of only one single cell that forms elongated tubes (non-articulated laticifers) that are often branched [7]. Thereby, the laticifers in the stems of most latex-bearing plants are most numerous close to the surface (e.g. the cortex) [8,9,10, personal observation], which is in accordance with the functions of the latex mentioned above, as this arrangement allows for an effective release of latex from injured plants. When considering these functions, also the time until the latex is completely coagulated (most latices then turn transparent) plays an important role. Whereas latex droplets of typical volume (about 10 µl) of most latex-bearing plants coagulate within about 20–30 minutes, others (e.g. *Campanula glomerata*) may coagulate within less than two seconds [11].

**Figure 1:** Laticifer types of plant species used in this study. Furthermore – as a comparison – the laticifer type of *Hevea brasiliensis* is included as well. Details of the systematic position of plant species, such as family and subfamily, are partially enclosed [7], [9], [32].

Most of the research on latex and latex-bearing plants has been conducted with regards to its use for the rubber processing industry. That is why mainly the latex of the Pará rubber tree (*Hevea brasiliensis*) has been examined in detail so far (see [12] for review). Other latex-bearing plants have mainly been examined because of their potential replacement of *H. brasiliensis* as a source of natural latex or to exploit new latex sources in regions where *H. brasiliensis* cannot be cultivated (e.g. [13]). However, little attention has been paid to the exploration of the coagulation mechanisms, let alone an insight into the possible diversity of different coagulation mechanisms of these plants so far. All coagulation mechanisms proposed in the current literature seem to be mainly chemically driven. In the case of *Hevea brasiliensis*, the coagulation is mediated by a protein which is released from burst vesicles into the plant latex due to a drop in pressure when the latex oozes out of a wound, and then cross-links rubber particles in the latex which leads to latex coagulation [12], [14], [15]. Wahler et al. [16] revealed that in the case of two *Taraxacum* species, both containing rubber particles, a different protein plays a major role in latex coagulation. For *Carica papaya* it was also proposed that the major component of latex clots during coagulation is protein [17], [18]. Therefore, this mechanism seems to differ profoundly from the above mentioned mechanisms, where rubber particles are the major components, as e.g. in *H. brasiliensis*. Instead of using unprocessed latex, in order to ease the examination of the key properties of interest (e.g. decelerated coagulation and thus a prolonged storage time), most latices have been processed or purified in scientific studies until now. However, in order to understand the processes taking place during latex coagulation *in planta*, the examination of natural, untreated latex is of major importance. This would not only help for a better understanding of the biological system, but could also be advantageous for the development of technical products beyond the classical rubber processing industry. For instance, the coagulation of plant latices may serve as a model for the development of biomimetic self-healing materials [19].

## Materials and Methods

### Plant material

The studies were carried out with one- to two-year old specimens of *Ficus benjamina* and about half a year old specimens of *Campanula glomerata*, *Euphorbia amygdaloides*, *E. characias* and *E. myrsinites* that were purchased from a local plant nursery. The plant species studied belong to the angiosperm families Moraceae, Campanulaceae and Euphorbiaceae, and represent only distantly related evolutionary lineages within the Eudicots (Figure 2).

**Figure 2:** Phylogenetic relationship of the plant species used in this publication. Species studied belong either to the families of Euphorbiaceae, Moraceae or Campanulaceae. The orders corresponding to the species studied are highlighted in bold. Adapted from [33].

### Particle size measurements (laser diffraction)

Particle size distributions of the plant latices were measured by laser diffraction with a particle size analyzer Malvern Mastersizer 2000 APA5001 (Malvern Instruments Ltd, Malvern, UK). For this purpose, fresh, uncoagulated latex was collected from freshly injured plants with a glass pipette and transferred to the dispersion unit filled with distilled water, until an obscuration between 9.4% and 13.6% was reached. The obscuration value depends on the sample concentration and quantifies the attenuation of the laser beam during the measurement. The ideal obscuration level for the measurements depends on the material density and range of particle sizes and - in general - is suggested by the manufacturer to be in the range between 3% and 30% (making sure that there is enough sample available to do the experiment). In order to disaggregate loose agglomerates of particles, 1 to 2 minutes of ultrasonic treatment was applied before measurements started. Detected particle sizes were converted by a computer model (Software Mastersizer 2000, Ver. 5.22, Malvern Instruments Ltd.: general purpose model, normal sensitivity) into a particle size distribution with a particle size range between 0.02 µm to 2000 µm (divided into 99 size classes, ensuring a sufficient amount of data points per graph). The particle volume within each size class was then given as the percentage of the total particle volume. The density of the fresh latex was needed for the calculation of the specific surface area. It was calculated by weighing a given volume of fresh latex droplets (collected with a pipette from the freshly injured plants; n = 10 for each plant species) and accounted 0.93±0.11 g cm^−3^ for *F. benjamina*, 1.12±0.09 g cm^−3^ for *E. amygdaloides*, 1.11±0.06 g cm^−3^ for *E. characias* and 1.06±0.10 g cm^−3^ for *E. myrsinites*.

### Particle visualisation

Images of plant latex and fresh plant tissue were taken with a cryo-scanning electron microscope Hitachi S-4800 (Hitachi High-Technologies Corp., Tokyo, Japan), equipped with a Gatan ALTO 2500 cryo-preparation system (Gatan Inc., Abingdon, UK). Temperatures were kept constantly at −140°C (prechamber) and −120°C (microscope). Cryo-scanning electron microscopy (Cryo-SEM) has been successfully used before to image little droplets on animal and plant surfaces [20], [21]. Fresh latex was collected by injuring the bark of the respective plants with a razor blade. Latex droplets were placed on a transfer device and immediately frozen in liquid nitrogen. Additionally to the fresh samples, plant latex droplets were collected as described above, but frozen in liquid nitrogen as soon as they were coagulated (i.e. as soon as they turned transparent).

For the examination of laticifers and latex particles *in planta*, up to 20 cm long parts of plants were frozen in liquid nitrogen. When frozen (covered with liquid nitrogen), segments of plant stems (from the lower part of the stem) and leaves from these stem segments were prepared and kept in liquid nitrogen until transferring them to the Cryo-SEM. If necessary, samples were heated up to −95°C in the prechamber to sublimate water from the sample surface. Subsequently, samples were sputter-coated with a 6–12 nm thick gold-palladium layer under an argon atmosphere. Images were taken at an acceleration voltage of 0.7–5 kV and a beam current of 10 microamperes (µA) using a secondary electron detector.

## Results

### Particle size measurements (laser diffraction)

The particle size distributions of the latex of the three *Euphorbia* species are similar to each other, while they markedly differ from that of the *Ficus benjamina* latex (Figure 3, Table 1). All three *Euphorbia* latices exhibit a narrow particle size distribution (minimum particle size class is 0.1 µm and maximum particle size class ranges between 0.3 µm and 0.51 µm) with one single peak between 0.17 µm and 0.2 µm. In contrast, even after applying various durations of ultrasonic treatment, the particle sizes of *F. benjamina* latex cover a wide range between 0.34 µm and 9.36 µm and reveal a bimodal distribution with peaks at 0.89 µm and 3.56 µm. Thus, the smallest particle sizes detected in *F. benjamina* latex are larger than the largest particle sizes found in *Euphorbia* latex (*E. characias*), or their particle sizes overlap only slightly (*F. benjamina* compared with both *E. amygdaloides* and *E. myrsinites*). Due to the larger particle sizes, the specific surface area of the *F. benjamina* latex amounts to only about 10% of that of the *Euphorbia* latices. With the method described above, the particle size distribution of *C. glomerata* latex could not be determined reproducibly as the fast coagulation is irreversible when using the untreated natural rubber. Even ultrasonic treatment could not resolve agglomerates at larger particle sizes.

**Figure 3:** Particle size distributions of the fresh latex of *Ficus benjamina* and of the three *Euphorbia* species. On the ordinate, the percentage of the volume of all particles within the respective size class related to the total volume (added volume of all particles in all size classes), is given. The latex was diluted in water and ultrasonic treatment was applied to dissolve loose aggregates before measuring. Fresh, uncoagulated latex of *Campanula glomerata* could not be measured, as it coagulates irreversibly before or while stirring in the dispersion unit. As a comparison, the particle size distribution of purified *H. brasiliensis* latex (data taken from Cornish & Brichta (2002) [27]) was added. The small inserted box shows the particle size distribution of *F. benjamina* latex when transformed to the number mode.

**Table 1:** Particle size distribution parameters of the fresh latex.

	Obscur. (%)	Conc. (%)	SSA (m^2^ g^−1^)	MinD (µm)	MinD (%)	MMT (µm)	MMT (%)	d (0.5) (µm)	MaxD (µm)	MaxD (%)
*Ficus benjamina*	13.6	0.0079	3.2	0.34	0.0064	3.56	11.4	3.01	9.36	0.12
*Euphorbia amygdaloides*	9.7	0.0033	29.6	0.10	0.0021	0.17	19.8	0.19	0.34	0.42
*Euphorbia characias*	9.9	0.0034	30.5	0.10	0.0015	0.17	20.2	0.18	0.30	3.94
*Euphorbia myrsinites*	9.4	0.0032	28.7	0.10	0.0009	0.20	18.6	0.20	0.51	0.01

The latex was diluted in water and ultrasonic treatment was applied before measuring. Obscur. = obscuration; Conc. = concentration (calculated from the Beer-Lambert law and given in % volume); SSA = specific surface area (total surface area of particles divided by their total weight); MinD = minimum particle size class detected - both the particle size [µm] and the corresponding volume [%] are given; MMT = maximum mode, where the maximum frequency distribution is reached - both the volume [%] and the corresponding particle size [µm], where this frequency was reached, are given; d (0.5) = median of the particle size distribution; MaxD = maximum particle size class detected - both the particle size [µm] and the corresponding volume [%] are given.

### Particle visualisation

Cryo-SEM studies comprised all three *Euphorbia* species, *F. benjamina* and *C. glomerata*. All particles in the latex are spherical and show only slight intraspecific variations in size. This not only holds for particles within the sample of a given specimen (see Figure 4), but also for samples from different specimens of the same plant species. The sizes of particles observed under the Cryo-SEM are in the range of sizes that were detected during laser diffraction measurements for all tested plant species. This does not only account for fresh, uncoagulated latex (Figure 4D for *F. benjamina* and – representative for all tested *Euphorbia* species – Figure 4A for *E. characias*), but also for coagulated latex (Figure 4B, E) and latex present in laticifers *in planta* (Figure 4C, F). Particles in the *F. benjamina* latex that are found in the central regions of latex droplets do not exhibit such a wide size distribution as detected using laser diffraction (Figure 3). However, structures that are larger in size were observed in the peripheral regions (e.g. the surface) of latex droplets (see below in the text and Figure 5). The latex particles observed *in planta* are not only of the same size, but also of the same shape as particles observed in fresh and coagulated latex, and are more densely packed in the *Euphorbia* laticifers than in those of *F. benjamina*. Furthermore, the diameter of laticifers in *E. characias* is larger compared to those observed in *F. benjamina*; especially in the laticifers of *E. characias*, almost no other cell content was observed besides latex particles, whereas in non-laticiferous cells no such particles were present. Also, in *C. glomerata* (Figure 6) and *F. benjamina*, particles were only observed in a few cells (i.e. the laticifers): - e.g. in Figure 7 for *F. benjamina* - in none of the cross-fractured cells (right picture margin in Figure 7) are latex particles present, while across the whole length of the longitudinally-fractured laticifer, particles of appropriate size can be seen (rest of Figure 7). Macroscopic observations that latex mainly oozes out in the peripheral region of the stem cross-section, when whole stems are penetrated, are confirmed by the Cryo-SEM studies: the laticifers are abundant in the peripheral region of the plant stems.

**Figure 4:** Cryo-SEM images of latex from *Euphorbia characias* and *Ficus benjamina*. Latex droplets were used both immediately after collecting (a, d) and as soon as they were coagulated (b including details at higher magnification, e). Pictures were taken from central regions of latex droplets (a, b, d, e). Latex particles of similar sizes can also be found *in planta* in laticifers of these plants (c including details at higher magnification, f).

**Figure 5:** Fractures in latex droplets of *Ficus benjamina*. The solid latex particles (e.g. black arrow in a) are not destroyed by fractures. Instead, fractures run around the latex particles (a, c). However, the larger and collapsed structures (e.g. white arrow in a) are divided by fractures (b) (Cryo-SEM images).

**Figure 6:** Laticifers in *Campanula glomerata* petiole (Cryo-SEM image).

**Figure 7:** Longitudinal fracture of a laticifer in a shoot axis of *Ficus benjamina*. Latex particles are abundant in the laticifer, but are absent in the surrounding cells (Cryo-SEM image).

Besides all the above mentioned spherical particles of the *F. benjamina* latex, the surface of those latex droplets additionally contains larger, collapsed structures (Figure 5). Particles with a size and shape comparable to particles in the central region of latex droplets are also found at or close to the surface (Figure 5A, C), whereas the collapsed structures are almost exclusively found right at the surface (Figure 5A, B), indicating a lower density at the droplet periphery. Differences in the stability between the small-sized latex particles and the larger (collapsed) structures become obvious upon closer examination of the propagation of cracks in their proximity. Cracks that develop during the fast freezing procedure of the latex in liquid nitrogen never penetrate the smaller particles. Instead, due to their high mechanical stability, cracks run around the particles without influencing their shape (Figure 5 C). In contrast, the larger collapsed structures typically become divided by the cracks (Figure 5 B) – cracks running around those larger structures were barely observed. In addition, these larger structures never exhibit smooth fracture planes after freeze fracturing of latex droplets or latex in laticifers as the smaller particles do (e.g. Figure 4D, F surface after freeze fracturing of a laticifer), but show considerably structured fracture surfaces instead.

## Discussion

The results presented here might provide the basis for a better understanding of the potential variety of latex coagulation mechanisms existing in plant species that have yet to be examined. Until now only the coagulation mechanisms of *Hevea brasiliensis* [12], [14], [15] and *Taraxacum* spp. [16] have been examined in detail, and a hypothesis for the coagulation of *Carica papaya* latex has been proposed [17], [18]. Additional studies using methods similar to those described in our paper concentrated on processed latices like preserved latex or purified latex particles (e.g. [22], [23], [24]), or on latices of more familiar plants (e.g. from *Hevea brasiliensis*, *Parthenium argentatum*, *Ficus elastica*, *Taraxacum* spp.), but without a comparative background (e.g. [23], [25]). To comprehend the variety and biological significance of latex composition and coagulation mechanisms existing in the ca. 40 plant families comprising latex-bearing plants, it is important to investigate the remaining unexamined or rather uncommon plant families and species. Additionally, one has to consider the functional mechanisms of latex coagulation from a more ‘biological point of view’ rather than to concentrate on the latex particles from an industry-oriented perspective.

For *Ficus benjamina*, *Euphorbia amygdaloides*, *E. characias* and *E. myrsinites*, the sizes of particles observed under the Cryo-SEM are in the range as observed during laser diffraction measurements for fresh, untreated, uncoagulated latex. The slight differences between particle sizes measured by laser diffraction and Cryo-SEM observation might be the effect of shrinkage or expansion of latex particles during freezing, depending on the molecular weight of the rubber [22]. The bimodal character of the particle distribution curve, obtained for *F. benjamina* using the laser diffraction method, is due to the fact that solid particles (smaller sizes) and collapsed structures (larger sizes) are present in the latex. Both types of structures were identified in the Cryo-SEM. A vesicular origin for the larger structures might be assumed due to their collapsed appearance in the Cryo-SEM, their low mechanical resistance to small stresses that caused small cracks in the latex (Figure 5), and due to their lower density if compared to other particles found in the latex.

In contrast, the smaller particles are mechanically much more stable in *F. benjamina* latex. Similarly, in other species belonging to the genus *Ficus*, and e.g. in *H. brasiliensis*, a similar mechanical stability and fracture behavior of the small latex particles were observed [22], [25]. The existence of both small particles and larger structures reveals similarities to the well-examined coagulation theory of *H. brasiliensis* latex, as first described by Gidrol *et* *al*., 1994 [14] (overview by D’Auzac *et al.*, 1995 [12]) and extended by Wititsuwannakul *et* *al*., 2008 [15]. According to this theory, coagulation is mediated by proteins stored in intact laticifers in vacuolar structures called lutoids. Upon injury of the laticifer, which is under high internal pressure of 8 bar or more ([26] and own measurements), these lutoids burst due to a fast pressure drop (to ambient pressure) and shear stresses within the rapidly discharging latex, and thus release their content. Some of the released proteins mediate a cross-linking between latex particles and lutoid fragments, as well as a latex particle-particle cross-linking, which leads to the coagulation of the latex. A particle size distribution considering only the first peak of the bimodal distribution curve for *F. benjamina* is very similar to that found for purified latex particles of *H. brasiliensis* [24], [27], where lutoids and its content are lacking (Figure 3). In fresh *H. brasiliensis* latex, lutoids may contribute 15 to 30% to the volume [12], [28] and have a diameter in the range of 2 to 10 µm [29], [30], which fits well with the second peak we observed for *F. benjamina* latex. Thus, not only the presence of the above mentioned particles and structures in *F. benjamina* latex, but also the comparability of their sizes to particles known from *H. brasiliensis* latex leads to the assumption that comparable coagulation mechanisms occur in these two species. Thereby, the quite small amount of collapsed structures in the latex compared to latex particles, as observed in the Cryo-SEM, is not contradictory to the fact that the second peak of the particle size analysis (i.e. at larger particle sizes) is much higher than the first one. Transforming the plot from ‘volume mode’ to ‘number mode’ (i.e., displaying the numbers of particles per particle size class on the ordinate instead of their total volume) reveals that the number of small particles (first peak) is much higher than that of the larger collapsed structures (second peak) (small box inserted in Figure 3).

Concerning particle sizes and other particle properties, *Euphorbia* spp. seem to have evolved a different coagulation mechanism. Here, even in the untreated fresh latex, no bimodal distribution curve of particle sizes was found. Instead, all three *Euphorbia* latices exhibit a sharp curve with peaks at very small particle sizes compared to the latices of most other plant species (e.g. *H. brasiliensis* or *F. benjamina*). Also in the literature, small particle sizes have been confirmed for other *Euphorbia* species (e.g. [22] for *E. lactiflua*). Furthermore, the particles are very densely packed in comparably large laticifers, whereas other cell content is much reduced compared to other latex-bearing plants. Upon injury, this leads to the release of a huge amount of particles being in close contact to each other with a specific surface area ten times that of the particles and structures in *F. benjamina* latex and still more than three times that of purified *H. brasiliensis* latex particles [24]. Thus, due to agglutination of the particle surfaces, a simple evaporation of water in the discharged latices of *Euphorbia* spp. has a much higher impact on the speed of coagulation compared to *H. brasiliensis* or *F. benjamina* latex. These facts lead us to hypothesize that the coagulation mechanism in *Euphorbia* spp. is not comparable to that of *H. brasiliensis* (which is based on chemical binding processes). Instead, it relies on physical cohesion processes and is mainly driven by the evaporation of water. The existence of different latex coagulation mechanisms among the plant kingdom is confirmed by findings from Bauer *et al.*, 2014 [31], who describe distinct differences between the latices of *F. benjamina* and *Euphorbia* spp. concerning their kinetics and rheological behavior during coagulation. They could show that coagulation of *Euphorbia* spp. latex is mainly evaporation-driven (enabling higher drying times and thus supporting a primary defensive role for their latex). In contrast, *F. benjamina* latex coagulates much faster involving a different process such as passive particle packing or active biochemical processes (ensuring a quick sealing and healing of the wound). Thus, our results support the findings of an evaporation-driven coagulation process for latices of *Euphorbia* spp. and an additional coagulation mechanism in the case of *F. benjamina* latex.

Unfortunately, particle size measurements yielded no reproducible results for the untreated natural latex of *Campanula* spp., as the very fast coagulation process makes it difficult to investigate. However, also in this case, not purified latex particles, but only the untreated latex could give reliable insights into the coagulation mechanism of this latex-bearing plant. Considering the speed of its coagulation, only a mechanism that cannot be compared to any mechanism proposed above might be likely.

In general, different latex coagulation mechanisms seem to not only be found in different plant families, but significant differences may also be found within species belonging to the same plant family. Although *H. brasiliensis* and *Euphorbia* spp. belong to the same plant family (Euphorbiaceae), their latices and their latex coagulation mechanisms show the most prominent differences. In contrast, the less evolutionary related plants, *H. brasiliensis* and *F. benjamina*, show remarkable similarities between their latices and the coagulation mechanism as investigated so far.

These findings allow us to hypothesize that there is a high selective pressure on the evolution of latices, and that in large latex bearing clades, as e.g. within the Euphorbiacean or the Moracean families, latex might possibly have evolved several times independently, or that at least markedly different latex types and coagulation mechanisms have evolved. Possibly this is triggered by various selective pressures acting on the plants and by different major functions of the latex in different habitats and different growth forms. For a better understanding of the composition and mode of functioning of latex as an important secondary plant metabolite, further comparative studies are necessary that will contribute to a better knowledge concerning the evolutionary origin and ecological significance of latices in the different latex bearing clades and plant species.

The methods used in this study might provide a rather quick and simple approach for a first characterization of latex composition and for reliable hypotheses on the potential coagulation mechanisms in a larger number and variety of latex-bearing plants. In combination with Cryo-SEM, the use of laser diffraction to determine particle sizes even exceeds the potential of monitoring the kinetics of rubber particle aggregation (as suggested by [24]) and thus might allow for fast interspecific comparisons of latex composition and potential coagulation mechanisms. These analyses can be checked later in selected species by much more sophisticated and time expensive detailed chemical analyses.
